# Application of Improved LSTM Algorithm in Macroeconomic Forecasting

This article has been retracted.

**DOI:** 10.1155/2021/4471044

**Published:** 2021-10-31

**Authors:** Shijun Chen, Xiaoli Han, Yunbin Shen, Chong Ye

**Affiliations:** ^1^School of Economics and Management, Tongji University, Shanghai 200092, China; ^2^School of Public Administration, Hainan University, Haikou 570228, China; ^3^School of Economics and Management, Fuzhou University, Fuzhou, Fujian 350108, China

## Abstract

From a macro perspective, futures index of agricultural products can reflect the trend of macroeconomy and can also have an early warning effect on the possible crisis and provide a reference for the government's economic forecast and macro control. Therefore, it is necessary to strengthen the research on early warning and prediction of agricultural futures price. For the prediction of futures price, there are two kinds of common models: one is the traditional classic time series model, and the other is the neural network model under the wave of artificial intelligence. This paper selects the 1976 closing data of agricultural futures index from January 10, 2012, to February 27, 2020, and uses the time series differential autoregressive integrated moving average model (ARIMA model) and long short-term memory model (LSTM model) to study this work, respectively, and compares the predicted effects of the two models in some metrics. Based on the predicted results of the two models, a simple trading strategy is established, and the trading effects of the two models are compared. The results show that the LSTM model has obvious advantage over ARIMA time series model in the price index prediction of agricultural futures market.

## 1. Introduction

In developed countries, commodity futures index has been running for decades and has become an important weathervane to reflect the trend of the financial market. However, compared with commodity futures market, as an important participant in the financial market, commodity futures are much less concerned than stocks and do not reflect their position in the national economic and social operation [1]. As a part of commodity futures, agricultural futures get less attention, so the research on the price prediction of agricultural futures will provide some reference for the existing academic research [2]. The price rise of agricultural products will increase consumer spending, which may lead to inflation. In the composition of consumer price index (CPI), the weight of food price accounts for about 1/3. The latest data showed that the CPI would rise by 2.9% in 2019, which is the highest growth rate since 2012. Among them, food affects the CPI rise by 3.82%, which has become the main force affecting the CPI rise. The most important raw materials for the food industry are agricultural products. Therefore, the impact of changes in the price of agricultural products on CPI is huge [3]. The research shows that the futures price index of agricultural products can reflect the real-time trend of CPI 3–6 months in advance. Therefore, from the macro level, the futures price index of agricultural products can reflect the macroeconomic trend, can also have an early warning effect on the possible crisis, and can provide reference for the government's economic forecast and macro control [4].

In addition, a single variety of agricultural futures cannot reflect the changes in the overall supply and demand relationship of the market, and the agricultural futures price index can overcome this limitation because it covers the main agricultural futures varieties [5]. From the micro level, for investors, the agricultural futures price index can reflect the overall trend of the agricultural futures market, help investors grasp the market trend in a more timely manner, adjust the proportion of investment, and provide reference for investors to carry out arbitrage trading of specific varieties, so as to maximize profits [6].

This paper is divided into five parts: the first part is the background of this work; the second part is the related work; it mainly analyses some current researches of ARIMA model and LSTM model and their application in agricultural futures market; the third part is the construction process for the improved LSTM model; it mainly introduces the model based on RNN model; the fourth part is the comparative experiment, comparing the forecasting effect of the LSTM and ARIMA models on the price index series of Zhengzhou commodity futures and Dalian commodity. The fifth part concludes this work and presents some findings.

## 2. Related Work

ARIMA model is one of the most common statistical models for time series prediction, which has been applied in various fields [7]. For example, Zhang et al. used least squares with forgetting factor for parameter estimation and a storm prediction algorithm for prediction. Through a large number of experiments, it was found that reducing forgetting factor can improve the performance of one-step prediction [8]. Han et al. used ARIMA method to establish electricity price forecasting and error forecasting models. In addition, they also collected historical data of electricity market and established daily average electricity price forecasting models based on ARIMA. The forecasting results of these models show that, compared with traditional electricity price forecasting methods, ARIMA model method is simple and clear, which significantly improves the forecasting accuracy [9]. Wang et al. collected the monthly incidence rate data in 1986∼2002 and used SPSS software to predict the incidence rate of notifiable infectious diseases by ARIMA model. The incidence rate of 2003 was predicted by the established model, and the predicted value was compared with the real value. The conclusion is that the ARIMA model can simulate the trend of the incidence rate of infectious diseases in time series and can predict the incidence rate in a more accurate way, providing a reference for the prevention and control of infectious diseases [10]. Yao et al. analysed Shenzhen's GDP from 1979 to 2006 and established ARIMA (1,2,2) model. Through the test of the model, it was found that the model can better predict Shenzhen's GDP, which can provide decision-making reference when Shenzhen sets economic development goals in the future [11]. Tafti et al. collected the gold price data from January 1973 to November 2010 and established the ARIMA model on this basis; the model effect is good [12]. Since the appearance of the LSTM model, many people have applied this model. Ramesh et al. established LSTM model. Compared with other original models, LSTM model has achieved the best level in standard evaluation so far, which fully demonstrates the powerful ability of LSTM in mining semantic information of text sequence [13]. Li et al. proposed an improved method based on LSTM network model based on the disadvantages of the current mainstream word segmentation methods. LSTM-based methods can achieve better results. For LSTM training time, GPU can greatly shorten the training time. In addition to word segmentation, LSTM method can also be extended to other natural language processings [14]. Parwez et al. constructed the LSTM model to fit and forecast the power load time series [15]. The power load data of a provincial power company is collected, and the LSTM model is used for simulation. The result proves that LSTM can predict the change of electric load in a short time. Hu et al. compared the three neural networks of BP, RNN, and LSTM, analysed whether the three models can be used, and compared the accuracy of the three models [16]. According to theoretical research and empirical analysis, it is found that, in the three models, LSTM neural network model can learn the existing stock market data, find the connection between the data, and use its unique selective memory function to dig out the internal law of stock price, so as to make a better short-term forecast [17]. However, in the research of agricultural products, LSTM model is rarely used. Hassib et al. obtained a large amount of price, weather, and other related data from multiple agricultural information platforms. According to the unique characteristics of agricultural product prices, long-term memory network > convolutional attention network > attention mechanism are combined, and neural network model integrating dual attention mechanism and long-term and short-term memory network is established [18]. It uses CNN model to extract features of influence factors of different components, adjust weights, and then send them to LSTM model to present the influence of time series and then send the results to attention mechanism to adjust weights and use the final results to predict agricultural product price index [19]. The results show that the model is superior to the traditional model in prediction accuracy. Similarly, LSTM model is rarely used in futures price forecasting. Talasila et al. established the arbitrage strategy model of ferrous metal futures market by using LSTM model and cointegration test method [20]. This paper collects the rebar futures listed in Shanghai Futures Exchange, coke futures listed in Dalian commodity exchange, and iron ore futures and makes an empirical study by using the arbitrage strategy model of ferrous metal futures market [21]. By comparing LSTM model, BP neural network, and convolution neural network, it is found that the LSTM-based model is the most effective [22]. Ait Hammou et al. selected the high-frequency data of main contracts of rebar varieties in commodity futures market from April to July 2017 to establish LSTM prediction model. The empirical analysis and back test results show that LSTM prediction model can better predict the short-term rise and fall trend of rebar varieties futures, indicating that it is suitable for high-frequency futures data [23]. As a relatively mature time series model, ARIMA model has a very wide range of applications in the economic and financial fields, but it is relatively less used in agricultural futures price forecasting. Therefore, this paper can explore the application of ARIMA model in agricultural futures market [24]. As an improved RNN model, LSTM model was first proposed [25]. Although it was put forward early, with the development of computer and the update of algorithm, it has not been widely developed until now. It belongs to a relatively new model, and few people use it in the futures price forecast of agricultural products or even in the futures price forecast. This paper can also provide exploratory help for the wider application of LSTM model [26–32].

### 2.1. Improvement of LSTM Model (1) Model Structure

The following figure shows the main structure of LSTM model. In this paper, we will simplify the network to the structure on the right side of the figure, so that we can describe and push LSTM in chronological order and visualize it, as shown in Figure 1.

### 2.2. Model Calculation Process

Generally speaking, the learning process of LSTM model can be summarized in three steps:

- It propagates forward and updates the output value generated by each node
- During back propagation, the accumulated residual gradually back propagates
- The gradient of each weight is calculated, the gradient decreases, and the weight of each node is corrected

Next, we will deduce the forward propagation and back-propagation formulas (1) to (3), and the forward propagation is calculated in chronological order:

(1) $$\begin{array}{c} a_{k}^{t}=\sum_{h=1}^{H}w_{hk}b_{h}^{t}, \end{array}$$

(2) $$\begin{array}{c} a_{h}^{t}=\sum_{i=1}^{1}w_{ih}x_{i}^{t}+\sum_{h^{\prime }=1}^{H}w_{h^{\prime }h}b_{h^{\prime }}^{t-1}, \end{array}$$

(3) $$\begin{array}{c} b_{h}^{t}=\theta_{h}\left(a_{h}^{t}\right). \end{array}$$

In the above formulas, letter *a* means the value of collection calculation. The superscript *t* indicates that the parameter value comes from node *t* at the time, letter *w* is the parameter connected between the nodes, and the specific node is determined by the subscript; *θ*_*h*_( ) is the activation function, and letter *b* means the value calculated by the activation function.

The third formula weights the activation function on the result of the second formula to obtain the result of the output layer. This also confirms our previous conclusion: there is a hidden layer in LSTM. The principle of back-propagation is the process of gradually transferring the accumulated residuals back from the last time point to correct the weights, as shown in the three following formulas:

(4) $$\begin{array}{c} \delta_{h}^{t}=\theta^{\prime }\left(a_{h}^{t}\right)\left(\sum_{k=1}^{K}\delta_{k}^{t}w_{hk}+\sum_{h^{\prime }=1}^{H}\delta_{h^{\prime }}^{t+1}w_{hh^{\prime }}\right), \end{array}$$

(5) $$\begin{array}{c} \delta_{j}^{t}\overset{\text{def}}{=}\frac{\partial ℒ}{\partial a_{j}^{t}}, \end{array}$$

(6) $$\begin{array}{c} \frac{\partial ℒ}{\partial w_{ij}}=\sum_{t=1}^{T}\frac{\partial ℒ}{\partial a_{j}^{t}}\frac{\partial a_{j}^{t}}{\partial w_{ij}}=\sum_{t=1}^{T}\delta_{j}^{t}b_{i}^{t}. \end{array}$$

The two summations in the form refer to the received residuals. The meaning of the above formula is to derive the residual values of two summation gradient descent and then correct the weight of each node.

### 2.3. Improved LSTM Model Construction

In the improved LSTM model, the hidden nodes are designed to be self-cycling. In this way, an error flow will be maintained in the memory cell, so that the information of a long time can be memorized, and the disappearance or explosion of the gradient can be effectively avoided.

Specifically, the special feature of LSTM model is the design of “door.” Each hidden node contains an information storage unit, and each storage unit contains three gates (logic unit): input gate, output gate, and forget gate. These three gates have different functions. The input gate and output gate are used to control the receiving and output of information, and the forget gate is used to control the selective forgetting of information in the storage unit. The function of parameters of input gate, output gate, and forget gate is only to set the weight at the connection between the storage unit and other units and will not be input to other neural units. Similar to RNN model, the weights of three gates corresponding to each storage unit are learned and generated in the training process.

### 2.4. Improved LSTM Model Calculation Process

For the improved LSTM model, it is controlled by forgetting gate, where *t* is the time and *sigmoi*  *d* is the unit number. Here we choose CC function, which can keep the weight between 0 and 1, as shown in the following formula:

(7) $$\begin{array}{c} f_{i}^{\left(t\right)}=\sigma \left(b_{i}^{f}+\sum_{j}U_{i,j}^{f}x_{j}^{\left(t\right)}+\sum_{j}W_{i,j}^{f}h_{j}^{\left(t-1\right)}\right), \end{array}$$

where *b*_*i*_^*f*^ represents the offset weight, *U*_*i*,*j*_^*f*^ represents the input weight, *W*_*i*,*j*_^*f*^ represents the cycle weight of the forgetting gate, *x*_*j*_^(*t*)^ represents the current input vector, and *h*_*j*_^(*t* − 1)^ represents the current hidden layer vector.

In the LSTM model, it is updated in the following way, including the self-loop weight of a condition; namely,

(8) $$\begin{array}{c} s_{i}^{\left(t\right)}=f_{i}^{\left(t\right)}s_{i}^{\left(t-1\right)}+g_{i}^{\left(t\right)}\sigma \left(b_{i}+\sum_{j}U_{i,j}x_{j}^{\left(t\right)}+\sum_{j}W_{i,j}h_{j}^{\left(t-1\right)}\right), \end{array}$$

where *b* is the weight of bias, *U* is the weight of input, and *W* is the cycle weight of forgetting gate. *g*_*i*_^(*t*)^ is an external input gate unit, which is similar to the update method of forgetting gate. The function expression is the same, except that it has its own parameters:

(9) $$\begin{array}{c} g_{i}^{\left(t\right)}=\sigma \left(b_{i}^{g}+\sum_{j}U_{i,j}^{g}x_{j}^{\left(t\right)}+{\sum_{j}W_{i,j}}^{g}h_{j}^{\left(t-1\right)}\right). \end{array}$$

When *sigmoi*  *d* unit is used as gate control, the output ore of each unit of LSTM model can also be closed through the output gate *q*_*i*_^(*t*)^; that is,

(10) $$\begin{array}{c} h_{i}^{\left(t\right)}=\tanh\left(s_{i}^{\left(t\right)}\right)q_{i}^{\left(t\right)}, \end{array}$$

(11) $$\begin{array}{c} q_{i}^{\left(t\right)}=\sigma \left(b_{i}^{0}+\sum_{j}U_{i,j}^{0}x_{j}^{\left(t\right)}+{\sum_{j}W_{i,j}}^{0}h_{j}^{\left(t-1\right)}\right), \end{array}$$

where *b*_*i*_^0^ is the weight of offset, *U*_*i*,*j*_^0^ is the weight of input, and *W*_*i*,*j*_^0^ is the cycle weight of forgetting gate.

### 2.5. Comparison Steps between LSTM and ARIMA Algorithm

Among them, for ARIMA time series model, this paper will use the auto ARIMA function in the forecast package of R language. For LSTM model, this paper will use Keras Library of Python language to build LSTM for training.

Firstly, we split the price index series into the first 70% training set and the last 30% testing set.

The training set is brought into ARIMA model. The mathematical expression of the AR(p) model is as follows:

(12) $$\begin{array}{c} y_{t}=\mu +\phi_{1}y_{t-1}+L+\phi_{p}y_{t-p}+\omega_{t}. \end{array}$$

The mathematical expression of the MA(*q*) model is as follows:

(13) $$\begin{array}{c} y_{t}=\mu +\omega_{t}+\theta_{t-1}\omega_{t-1}+L+\theta_{q}\omega_{t-q}. \end{array}$$

The formula of the model is shown as follows:

(14) $$\begin{array}{c} \nabla^{d}y_{t}=\mu +\phi_{1}y_{t-1}+L+\phi_{p}y_{t-p}+\omega_{t}+\theta_{1}\omega_{t-1}+L+\theta_{q}\omega_{t-q}, \end{array}$$

where *d* denotes the difference times and other coefficients have the same meaning as AR(*p*) and MA(*q*).

It is not difficult to see that if *p* = 0, *ARIMA* model is *MA*(*q*) model; and if *q* = 0, *ARIMA* model is AR(p) model.

Next, we will introduce the training and testing process of LSTM model as follows: first-order difference is a common skill in processing time series data, and the time series after difference is transformed into (*x*, *y*) data pairs. The data pair is divided into training data pair and testing data pair one by one. Standardizing the independent variable *X* of training data pair and testing data pair to [−1, 1] interval is a common normalization operation, which is beneficial to LSTM training.

Build LSTM model and train it. The “rolling prediction” of the testing set is carried out to obtain the estimated value of the “after difference” sequence. According to the *y* value, the estimated value of the test sequence can be obtained. If you choose the hyperparameters of the LSTM model, you can bring the first 70% of the training set and validation set into the above process to get the result.

## 3. Results and Discussion

### 3.1. Data Acquisition and Processing

Research on the trend prediction of price index is widely used in the stock market. However, we can also focus on the futures market. As a trading market with higher risk than the stock market, futures market is also concerned by many professional investors. CAFI is the monitoring center of agricultural futures index. For each futures market, the time series data of futures price index includes six attributes. In the following empirical analysis, we select the “closing price” as the feature of time series and use ARIMA time series model and LSTM to predict the “closing price” of the next trading day. The training of the improved LSTM model needs supervised data, that is, the paired data of “independent variable and dependent variable.” Therefore, for a time series data, it is necessary to transform it into supervisory data first. For example, if the value of a certain time in the series is regarded as the dependent variable to be estimated, then the past observation will be regarded as the independent variable for the prediction of that time. Firstly, the two-dimensional coefficient matrices *A*_1_ and *A*_2_ of *N* × *N* are generated randomly. Then *Y*_0_ ∈ exp(*N*(0, *l*)) is generated randomly; the appropriate *a* and *b* values are selected. Here we set *a*=1 and *b*=0.5.

For each period from 1 to SS, it is according to the following formula:

(15) $$\begin{array}{c} Y_{t}=A_{1}Y_{t-1}+A_{2}\left(a\max\left(Y_{t-1},b\right)\right)+\varepsilon_{t}. \end{array}$$

Figure 2 shows the original data of the improved LSTM model and the changes after the training process.

The red line, green line, and blue line are all VAR models; the green line is the estimation model with 4 lags, the red line is the estimation model with 3 lags, the blue line is the estimation model with 2 lags, and the yellow line is the LSTM enhancement model. It can be seen from the figure that the training loss of the VAR model during the training process is larger than that of the new model, and the fluctuation range is also greater. After the training times of the new model, the training loss almost stagnates and decreases, but this is mainly due to the training loss of the new model. The initial level is quite low, and a larger drop requires more training; and the training loss fluctuates little throughout the training process, indicating that the new model is not only better in performance but also more robust. After several rounds of training, the authors found that the training loss change graph drawn after each training has the above characteristics.

The performance of the trained model on the test set is more important. In order to measure the performance of the new model and the three control models on the testing set, repeat the above data and train 5000 rounds of simulation model (simulation data is regenerated in each round, and training starts with randomly generated parameters) and training in each round. After completion, test the model on the test set generated in this round. From this, the test loss of 5000 groups of models on the testing set can be obtained. Round the test loss to 2 decimal places to get the distribution of testing loss of each model on the testing set. The distribution is shown in Figure 3.

### 3.2. Evaluation Index and Prediction Method

The root mean square error is used to measure the effectiveness of the prediction model. The calculation formula is as follows [33–39]:

(16) $$\begin{array}{c} \text{RMSE}=\sqrt{\frac{1}{N}\sum_{i=1}^{N}{\left(x_{i}-{\hat{x}}_{i}\right)}^{2}}. \end{array}$$

In the scene of time series prediction, when we use the known time series to train the time series prediction model, with the time moving forward, the current time is farther and farther away from the known time series, and the accuracy of time series prediction will be lower and lower. Therefore, we use the “forward model verification” method for prediction; that is, when a new observation is obtained at each time, the new observation is input into the time series prediction model for updating, which is called “rolling prediction.” In the empirical analysis of this paper, we first use the first 70% of the data series for training and then do the above “rolling prediction” for the last 30% of the exponential series. Under the premise of fixed model super parameters, we update the time series prediction model with new observations at each time and then predict the value of the next time.

### 3.3. Comparative Experiment between ARIMA Time Series Model and Improved LSTM Model

The empirical analysis of this paper will carry out the comparative test of ARIMA time series model and LSTM and compare the forecasting effect of the two methods on six futures price index series. Experimental results of LSTM model are shown in the figure below, where the blue solid line is the real observation value of the test sequence. The red-dotted line is the prediction value of LSTM model: the experimental results of ARIMA and LSTM prediction models are shown in Figures 4to 7, where the blue solid line is the real observation value of the test sequence, and the red-dotted line is the prediction value of ARIMA time series.

It can be seen that the fluctuation of Dalian commodity index predicted by ARIMA model is basically the same as the real value. Compared with the real value, the fluctuation of the predicted value has a delay of 3–4 days. The peak of Dalian commodity index appears on October 31, 2019, and the lowest point appears on December 20, 2019, and the fluctuation is very intense. The peak and the lowest point of the predicted value appear 4 days later than the real value.

The predicted value of ARIMA's Zhengzhou commodity index is 3–4 days later than the real value. The highest point of Zhengzhou commodity index appears on January 2, 2019. Before January 2, 2019, the commodity index shows a gradual upward trend, and, after January 2, 2019, the commodity index shows a gradual downward trend.

The volatility of LSTM's Dalian commodity index is basically the same as the real value, but the overall trend is low. Dalian commodity index presents the characteristics of violent fluctuations, with the highest point on January 2, 2020, and the lowest point on December 20, 2019. Compared with the real value, the predicted value obtained by LSTM is delayed by 4 days, and the commodity index is lower than the highest point and the lowest point.

The prediction results of ARIMA time series model and LSTM model on six futures price index series are summarized in Table 1.

It can be found from the table that the improved LSTM model has obvious advantages over ARIMA time series model.

## 4. Conclusion

Because grain prices have fluctuated greatly in the past two years, the majority of farmers have been affected. For investors, greater profits can be obtained by reasonably matching the variety and quantity of futures. In Europe and the United States and other developed countries, commodity futures index has been running for decades and has become an important weathervane to reflect the trend of the financial market. However, compared with commodity futures market, as an important participant in the financial market, commodity futures are much less concerned than stocks and do not reflect their position in the national economic and social operation. As a part of commodity futures, agricultural futures get less attention, so the research on the price prediction of agricultural futures will provide some reference for the existing academic research. Therefore, it is necessary to strengthen the research on early warning and prediction of agricultural futures price. This paper selects the 1976 day closing data of agricultural futures index from January 10, 2012, to February 27, 2020, and uses ARIMA model and LSTM model to build models, respectively. By comparing the RMSE of the two models, the paper compares the prediction effect of the two models. Compared with ARIMA time series model, the improved LSTM model has obvious advantages.

## Figures and Tables

**Figure 1:** LSTM unfolding structure.

**Figure 2:** Data sketch and training process changes.

**Figure 3:** The distribution of training loss.

**Figure 4:** Comparison of ARIMA model's forecast value and real value of Dalian commodity index.

**Figure 5:** Comparison of ARIMA model's forecast value and real value of Zhengzhou commodity index.

**Figure 6:** Comparison of Dalian commodity price index predicted by improved LSTM model with real value.

**Figure 7:** Comparison of Zhengzhou commodity price index predicted by improved LSTM model with real value.

**Table 1:** Two models of commodity market index forecast results.

Futures market	RMSE	
	ARIMA	LSTM
Dalian	5.637	2.6378
Zhengzhou	6.1173	2.1287

## Data Availability

The data used to support the findings of this study are available from the corresponding author upon request.
